# High Prevalence of *bla*_NDM_ Variants Among Carbapenem-Resistant *Escherichia coli* in Northern Jiangsu Province, China

**DOI:** 10.3389/fmicb.2018.02704

**Published:** 2018-11-13

**Authors:** Ruru Bi, Ziyan Kong, Huimin Qian, Fei Jiang, Haiquan Kang, Bing Gu, Ping Ma

**Affiliations:** ^1^Medical Technology School, Xuzhou Medical University, Xuzhou, China; ^2^Jiangsu Provincial Center for Disease Control and Prevention, Nanjing, China; ^3^Department of Laboratory Medicine, Affiliated Hospital of Xuzhou Medical University, Xuzhou, China

**Keywords:** carbapenem, *Escherichia coli*, *bla*_NDM_ variants, diversity, plasmid

## Abstract

The continuous emergence of carbapenem-resistant *Escherichia coli* (CRECO) presents a great challenge to public health. New Delhi metallo-lactamase (NDM) variants are widely disseminated in China, so the research on the prevalence and transmission of diverse *bla*_NDM_ variants is urgently needed. In the present study, 54 CRECO isolates were collected from 1,185 *Escherichia coli* isolates in five hospitals in Northern Jiangsu Province, China from September 2015 to August 2016. Antimicrobial susceptibility tests, PCR detection of resistance determinants, multi-locus sequence typing (MLST) and pulsed-field gel electrophoresis (PFGE) were performed to characterize these strains. Plasmid conjugation experiments were carried out to determine the transferability of resistant genes from selected isolates. PCR-based replicon typing (PBRT), S1 nuclease-PFGE, and Southern blotting were conducted for plasmid profiling. Carbapenemase genes were detectable in all CRECO isolates, among which thirty-one CRECO isolates were found to carry *bla*_NDM−5_ (54.7%), while, *bla*_NDM−1_, *bla*_NDM−7_, *bla*_NDM−4_, *bla*_NDM−9_, and *bla*_KPC−2_ were identified in 14, five, two, one, and one isolates, respectively. MLST results revealed 15 different STs and four new STs were first reported to be linked with NDM-producing isolates. PFGE typing showed that no more than two isolates with the same ST appeared to the same band pattern except three ST410 isolates. Twenty-six selected NDM-producing isolates were successfully transferred to *E. coli* J53 by conjugation experiments. Notably, 50.0% (13/26) of *bl*a_NDM_ variants were found to be carried by ~55 kb IncX3 plasmid. Our study reported a high prevalence of *bl*a_NDM_ variants, especially *bla*_NDM−5_, in Northern Jiangsu province, China. Diverse *bla*_NDM_ variants were mainly carried by ~55 kb IncX3 plasmids, suggesting that the fast evolution and high transferability of this kind of plasmid promote the high prevalence of *bla*_NDM_ variants. Therefore, large-scale surveillance and effective infection control measures are also urgently needed to prevent diverse *bla*_NDM_ variants from becoming epidemic in the future.

## Introduction

Carbapenem, a β-lactam that is highly potent against Gram-negative bacteria, has been recognized as a last resort for treating of infections caused by multidrug-resistant bacteria. However, the increasing number of carbapenem-resistant *Enterobacteriaceae* (CRE) is unexpected despite infection control efforts, and it poses a great challenge to clinic (Zilberberg and Shorr, 2013). Carbapenem resistance is predominantly attributed to the presence of carbapenemases, among which Class A (*bla*_KPC_), Class B (*bla*_NDM_*, bla*_VIM_*, bla*_IMP_), and Class D (*bla*_OXA−48_) types are most common for *Enterobacteriaceae* (Walsh, 2010; Albiger et al., 2015). An emerging carbapenemase, New Delhi metallo-lactamase (NDM), was first reported in a Swedish patient with a hospitalization history in India, it exhibited resistant to all β-lactams except for monobactams, and has great potential to cause global health crisis (Yong et al., 2009). Initially, *bla*_NDM_ gene was endemic to India subcontinent and NDM-producing isolates tested worldwide have geographical links with these high prevalence areas. However, an increasing number of regions worldwide have reported that patients with *bla*_NDM−_positive isolates have never been abroad, indicating that *bla*_NDM_ genes are also associated with some special clones (Leverstein-Van et al., 2010).

In China, since the first report of *bla*_NDM_ gene in four carbapenem-resistant *Acinetobacter baumannii* isolates (Chen et al., 2011), increasing *Enterobacteriaceae* have been identified as carriers of the *bla*_NDM_ gene. *Escherichia coli*, an important member of *Enterobacteriaceae*, are often spread globally through some epidemiological lineages. Although the prevalence of NDM-producing CRE strains is low, outbreaks caused by *bla*_NDM_-positive isolates have been identified in several regions of China, indicating high transferability of the *bla*_NDM_ gene and the severity of infections caused by *bla*_NDM−1_-positive organisms (Wang et al., 2014; Jin et al., 2015; Yu et al., 2016). Furthermore, Kaase et al. (2011) first reported a novel *bla*_NDM_ variant, *bla*_NDM−2_, which differs by one amino acid substitution (Pro28Ala) from *bla*_NDM−1_, and the subsequent discovery of other *bla*_NDM_ variants highlights the rapid evolution of this multi-drug resistance gene. In 2012, the NDM enzyme reservoir, India, first reported diverse *bla*_NDM_ variants among *Enterobacteriaceae* and *bla*_NDM_ variants exhibited higher minimum inhibitory concentration (MIC) levels of carbapenem compared with *bla*_NDM−1_ (Rahman et al., 2014). Although the *bla*_NDM_ gene is continuously recoverable in China, data on the prevalence and characteristics of *bla*_NDM_ variants among *Enterobacteriaceae* are still needed for preventing its transmission. Notably, a study conducted by Hu et al. (2017) have discovered that various species of bacteria harbored several kinds of *bla*_NDM_ variants in China, which were mainly carried by diverse plasmids with different sizes. In the present study, we reported a high prevalence of *bla*_NDM_ variants among *E. coli* from five hospitals in Northern Jiangsu Province, China. Moreover, these diverse *bla*_NDM_ variants were mainly located on the same plasmid.

## Materials and methods

### Study design

From September 2015 to July 2016, five hospitals (two in Xuzhou, two in Suqian, and one in Lianyungang) in Northern Jiangsu Province of China collected 1,185 *E. coli* isolates to examine the prevalence and molecular epidemiology of carbapenem-resistance isolates. Initial species identification and antimicrobial susceptibility testing was performed by the Vitek 2 system (bioMe'rieux, France) and MALDI-TOF MS (Bruker Microflex LT, Bruker Daltonik GmbH, Bremen, Germany) according to the manufacturer's instructions.

### Antimicrobial susceptibility testing

Initial susceptibility testing was examined by Vitek 2 system. Further MICtesting was conducted by agar dilution method for cefoxitin, ceftriaxone, ceftazidime, cefepime, aztreonam, amikacin, ciprofloxacin, tigecycline, and piperacillin/tazobactam. The MICs of imipenem, meropenem, and ertapenem were determined by E-tests. For colistin, MIC values were tested by broth microdilution method. The agar dilution method and E-test were performed according to the standard Clinical and Laboratory Standards Institute guideline (M100-S26) (CLSI, 2017). The breakpoints of Food and Drug Administration (FDA) and European Committee on Antimicrobial Susceptibility Testing were used for tigecycline and polymyxin, respectively.

### Molecular detection of resistance genes

DNA templates were prepared by alkaline lysis method using the kit (MoBio, USA). Carbapenemase genes (*bla*_KPC_ *bla*_NDM_, *bla*_SME_*, bla*_GES_*,bla*_VIM_*, bla*_IMP_, and *bla*_OXA−48_) (Senda et al., 1996; Queenan et al., 2000; Poirel et al., 2004; Endimiani et al., 2008; Yang et al., 2012; Pereira et al., 2015; Al-Agamy et al., 2017), extended spectrumβ-lactamase genes (*bla*_SHV_*, bla*_TEM_*, bla*_CTX−M−1group_*, bla*_CTX−M−2group_*, bla*_CTX−M−8group_, and *bla*_CTX−M−9group_) (Schmitt et al., 2007; Yu et al., 2007), and plasmid-mediated AmpC genes(*bla*_ACC_*, bla*_FOX_*, bla*_MOX_*, bla*_DHA_*, bla*_CIT/SPM_, and *bla*_EBC_) (Pérez-Pérez and Hanson, 2002) were examined by PCR. *E. coli* ATCC25922 was used for the quality control. Positive amplifications were subject to Sanger sequencing (GENEWIZ Company, Suzhou, China).

### PFGE and MLST

Molecular typing of 54 NDM-producing *E. coli* isolates was performed by pulsed-field gel electrophoresis (PFGE). The plugs containing genomic DNA were prepared according to the procedure described by Pereira et al. (2015). The DNA fragments digested with restriction endonuclease *XbaI* (TaKaRa Biotechnology, Dalian, China) were separated by PFGE on 1% SeaKem Gold agarose (Lonza, Rockland, ME, USA) using the CHEF Mapper XA PFGE system (Bio-Rad, USA) for 18 h at 14°C. The electrophoretic switch times were 6.8–35.4 s. *Salmonella* H9812 was used as reference marker. Dice coefficients was used to calculate the similarity of PFGE patterns. Dendrograms were constructed by the unweighted pair group method with arithmetic averages (UPGMA) using BioNumerics software version 5.10. Isolates were categorized to be of the same cluster when their dice similarity index was ≥85%. Multi-locus sequence typing of *E. coli* was conducted by PCR as previously described (Wirth et al., 2006). The allelic profiles and sequence types were identified by amplifying and sequencing the seven housekeeping genes (*adk, fumC, gyrB, icd, mdh, purA, recA*) according to the reference website (https://enterobase.warwick.ac.uk/species/index/ecoli). A minimum spanning tree of 54 *bla*_NDM_-positive isolates was also constructed by BioNumerics software version 5.10.

### Conjugation assay

The conjugation experiment was implemented by mix broth mating among 26 selected isolates. The donor (clinical strains harboring the *bla*_NDM_ gene) and recipient (sodium azide-resistant *E. coli* J53) were mixed and cultured in broth at 37°C overnight. The transconjugants were selected on MH agar with sodium-azide (180 μg/mL) and imipenem (1 μg/mL). Initial species identification was conducted by Vitek MS system. Transformants were regarded as transconjugants when it exhibited resistance to carbapenem and harbored the *bla*_NDM_ gene.

### Plasmid analysis

Twenty-six selected isolates, including *bla*_NDM_-_5_ and *bla*_NDM_-_1_ gene with different STs from the aforementioned five different hospitals and all *bla*_NDM_-_4_ (one isolates was lost in transit), *bla*_NDM_-_7_, and *bla*_NDM_-_9_-positive isolates, were subjected to further plasmid analysis. Incompatibility groups of plasmids extracted from transconjugants were determined by PCR-based replicon typing as described previously (Carattoli et al., 2005; Johnson et al., 2012). S1-PFGE and Southern blotting were conducted to isolate and locate resistance plasmids. Briefly, the gel plugs embedded with *bla*_NDM_-positive isolates were digested with S1 nuclease (TaKaRa Biotechnology, Dalian, China) and linear plasmids were separated by CHEF-Mapper XA PFGE system (Bio-Rad) as described above. The universal primers (F: GAAGCTGAGCACCGCATTAG; R: GGGCCGTATGAGTGATTGC) were used for probe synthesis. The plasmid DNA were transferred to positive-charged nylon membranes (Millipore, USA), and DIG-labeled *bla*_NDM−_specific probe served to hybridize plasmids according to the instructions of the DIG High Prime DNA Labeling and Detection Starter Kit (Roche, USA).

## Results

### Clinical data and prevalence of carbapenemase genes among CRECO

A total of 54 (4.56%, 54/1185) non-duplicate *E. coli* isolates that exhibited resistance to imipenem or meropenem were obtained from five hospitals in Northern Jiangsu Province, China. The Affiliated Hospital of Xuzhou Medical University (Hosptial A, *n* = 18), the Children's Hospital of Xuzhou (Hosptial B, *n* = 13), the People's Hospital of Suqian (Hosptial C, *n* = 11), the First People's Hospital of Suqian (Hosptial D, *n* = 6), and the Second People's Hospital of Lianyungang (Hosptial E, *n* = 6) were included. Among 54 CRECO isolates, 53 (98.1%, 53/54) were found to be *bla*_NDM_-positive and 1 was *bla*_KPC−2_-positive. Interestingly, five different *bla*_NDM_ variants were identified in this collection (Figure 1). Among them, the *bla*_NDM−5_ was the prevailing variant, accounting for 58.5% (31/53) of *bla*_NDM_-positive isolates, followed by *bla*_NDM−1_ (26.4%, 14/53). Moreover, *bla*_NDM−7_, *bla*_NDM−4_, and *bla*_NDM−9_ genes were also identified in 5, 2, and 1 isolates, respectively. NDM variations in amino acid substitutions at various positions are shown in Table 1. The distribution of the *bla*_NDM_ variants in hospitals is depicted in Figure 1.

**Figure 1:** The distribution of *bla*_NDM_ variants among different hospitals. Hospital A, the Affiliated Hospital of Xuzhou Medical University; Hospital B, the Children's Hospital of Xuzhou; Hospital C, the People's Hospital of Suqian; Hospital D, the First People's Hospital of Suqian; Hospital E, the Second People's Hospital of Lianyungang.

**Table 1:** Amino acid substitutions of initially reported NDM variants.

**NDM-type**	**Val 88**	**Asp 130**	**Glu 152**	**Met 154**	**Isolates**	**Country**	**Tourism history**	**GenBank accession no**.
NDM-1	–	–	–	–	*K. pneumoniae, E. coli*	Sweden	India	FN396876
NDM-4	–	–	–	Leu	*E. coli*	Cameroon	Pakistan	JQ348841
NDM-5	Leu	–	–	Leu	*E. coli*	UK	India	JN104597
NDM-7	–	Asn	–	Leu	*E. coli*	UK	Spain	JX262694
NDM-9	–	–	Lys	–	*K. pneumoniae*	China	No	KC999080

### Antimicrobial susceptibility patterns and prevalence of additional resistance genes of NDM-producing CRECO

Fifty-three NDM-producing CRECO isolates were resistant to all cephalosporins (cefoxitin, ceftriaxone, ceftazidime, and cefepime) and enzyme inhibitors (piperacillin/tazobactam) but remained susceptible to colistin and tigecycline. The resistance rates to aztreonam, amikacin, and ciprofloxacin were 84.9, 22.6, and 92.4%, respectively. As shown in Table 2, among 31 *bla*_NDM−5_-positive isolates, 93.5% were resistant to ciprofloxacin, 74.2% to aztreonam, and 32.2% to amikacin. Resistance to aztreonam and ciprofloxacin were 85.7 and 92.9% among 14 *bla*_NDM−1_-producing isolates and were susceptible to amikacin. As for *bla*_NDM−7_-positive isolates, susceptibility was only found for amikacin. The *bla*_NDM−4_ and *bla*_NDM−9_ isolates were resistant to all antibiotics tested in this study except for colistin and tigecycline. One *bla*_KPC−2_-positive isolate was resistant to amikacin, colistin, and tigecycline. Molecular features revealed that most CRECO isolates carried the ESBLs gene, AmpC gene, or both. Overall, *bla*_CTX−M_*, bla*_SHV_, and *bla*_TEM_ were identified in 42, 11, and 32 isolates, respectively. *bla*_CTX−M_-_15_ was the most common ESBLs gene in our study, accounting for 26.4% followed by *bla*_CTX−M_-_55_ (*n* = 9), *bla*_CTX−M_-_65_ (*n* = 8), *bla*_CTX−M_-_14_ (*n* = 8). *bla*_CTX−M_-_64_ (*n* = 1), *bla*_CTX−M_-_90_ (*n* = 1), and *bla*_CTX−M_-_123_ (*n* = 1). All *bla*_TEM_ positive isolates were identified as *bla*_TEM−1_. Moreover, 6 *bla*_CMY−2_, 5 *bla*_CMY−42_, and 1 *bla*_DHA−1_ were also identified.

**Table 2:** Antimicrobial susceptible patterns of NDM-producing *Escherichia coli*.

**Antibotic**	**Total (*****n*** = **53)**		**NDM-5 (*****n*** = **31)**		**NDM-1 (*****n*** = **14)**		**NDM-7 (*****n*** = **5)**		**NDM-4 (*****n*** = **2)**		**NDM-9 (*****n*** = **1)**	
	**S (%)**	**R (%)**	**S (%)**	**R (%)**	**S (%)**	**R (%)**	**S (%)**	**R (%)**	**S (%)**	**R (%)**	**S (%)**	**R (%)**
IMP	0.0	100.0	0.0	100.0	0.0	100.0	0.0	100.0	0.0	100.0	0.0	100.0
MEP	0.0	100.0	0.0	100.0	0.0	100.0	0.0	100.0	0.0	100.0	0.0	100.0
ETP	0.0	100.0	0.0	100.0	0.0	100.0	0.0	100.0	0.0	100.0	0.0	100.0
FOX	0.0	100.0	0.0	100.0	0.0	100.0	0.0	100.0	0.0	100.0	0.0	100.0
CRO	0.0	100.0	0.0	100.0	0.0	100.0	0.0	100.0	0.0	100.0	0.0	100.0
CAZ	0.0	100.0	0.0	100.0	0.0	100.0	0.0	100.0	0.0	100.0	0.0	100.0
FEP	0.0	100.0	0.0	100.0	0.0	100.0	0.0	100.0	0.0	100.0	0.0	100.0
ATM	15.1	81.1	22.6	74.2	7.1	85.7	0.0	100.0	0.0	100.0	0.0	100.0
AMK	75.4	22.6	67.7	32.2	92.9	0.0	60.0	40.0	0.0	100.0	0.0	100.0
CIP	5.7	92.4	6.5	93.5	7.1	92.9	0.0	80.0	0.0	100.0	0.0	100.0
TZP	0.0	100.0	0.0	100.0	0.0	100.0	0.0	100.0	0.0	100.0	0.0	100.0
TGC	100.0	0.0	100.0	0.0	100.0	0.0	100.0	0.0	100.0	0.0	100.0	0.0
COL	100.0	0.0	100.0	0.0	100.0	0.0	100.0	0.0	100.0	0.0	100.0	0.0

*IMP, imipenem; ETP, ertapenem; MEP, meropenem; PB, colistin; TGC, tigecycline; ATM, aztreonam; FOX, cefoxitin; FEP, cefepime; CA, ceftazidim; CRO, cefatriaxone; YZP, piperacillin/tazobactam; AMK, amikacin; CIP, ciprofloxacin*.

### Molecular typing of CRECO

A total of 15 STs were identified in 54 CRECO isolates (Figure 2). Among 53 *bla*_NDM_-producing isolates, ST167 was the most prevalent, accounting for 35.8% (19/53), followed by ST410 (16.9%, 9/53), ST617 (13.2%, 7/53), ST405 (5.6%, 3/53), ST155 (3.8%, 2/53), ST156 (3.8%, 2/53), ST361 (3.8%, 2/53), and ST2659 (3.8%, 2/53). ST90, ST224, ST46, ST648, ST2376, and ST2083 were identified in one isolate. ST167 and ST617 are different by one allele and both correspond to clonal complex CC10. Moreover, ST410 and ST90 belong to clonal complex CC23. One KPC-2-producing isolate belong to ST131. PFGE typing revealed that no more than two isolates with the same ST type appeared to the same band pattern except for three ST410 isolates from hospital B (Figure 3). Surprisingly, the two isolates (E11 and E28) from hospital A and B shared the same patterns, indicating the occurrence of cross-transmission between hospitals.

**Figure 2:** Minimum spanning tree of 54 CRECO isolates from different hospitals.

**Figure 3:** Dendrogram of PFGE profiles of 54 CRECO isolates. The UPGMA algorithm was used to construct dendrogram based on the dice similarity coefficient. Isolates were categorized to be of the same cluster when their dice similarity index was ≥ 85%.

### Characteristic of plasmids harboring the *bla*_NDM_ gene

All of plasmids haboring *bla*_NDM_ gene from 26 selected CRECO isolates were successfully transferred to *E. coli* J53, and transconjugants exhibited resistance to carbapenem, cephalosporins and enzyme inhibitors (Table 3). As shown in Figure 4, S1-PFGE and Southern blotting revealed that all *bla*_NDM−5_ genes were located on the same size (~55 kb) plasmids, which was associated with IncX3 (*n* = 5), IncFI (*n* = 3), IncFII (*n* = 1), and untypeable replicon (*n* = 3). The *bla*_NDM−1_ genes were carried by 55~210 kb plasmids, including IncX3 (*n* = 5), IncFI (*n* = 1), and IncFII (*n* = 1) replicon types. Among five *bla*_NDM−7_ positive isolates, four harbored ~55 kb IncX3 plasmids with DIG-labeled *bla*_NDM−7_, and the remaining one was carried by ~110 kb IncFI plasmid. The *bla*_NDM−4_ and *bla*_NDM−9_ genes were located on ~55 kb IncX3 and ~110 kb IncI1 plasmids, respectively. Surprisingly, E5 isolates harbored three *bla*_NDM−5−_positive plasmids of ~55, ~105, and ~320 kb in size, suggesting high insertion efficiency of the *bla*_NDM_ gene. Further plasmid sequencing from E5 isolates revealed that the respective GenBank accession numbers for ~55 and ~105 kb plasmids were NC_022740.1 and AP018144.1, however, the nucleotide sequences of ~320 kb plasmid could not be completely obtained.

**Table 3:** Antimicrobial susceptible patterns and characteristics of 26 selected NDM-producing *Escherichia coli* (μg/mL).

**Isolates**				**Antimicrobial susceptible**							**Hospital**			**Carbapenemase**	**MLST**	**Imp and size (kb)**	
	**ETP**	**IMP**	**MEP**	**FOX**	**CRO**	**CAZ**	**FEP**	**ATM**	**AMK**	**CIP**	**TZP**	**TGC**	**PB**				
E5	>32	32	>32	>256	>256	>256	>256	>256	>256	32	>256	0.5	0.5	A	NDM-5	ST167	X3/55^a^, FII/105^b^,UT/320
E5-J53	8	2	4	>256	>256	>256	16	64	0.5	≤ 0.06	256	0.25	0.25				
E7	8	8	4	>256	256	>256	32	16	>256	64	128	0.25	0.5	A	NDM-5	ST224	FII/55
E7-J53	4	2	4	>256	256	>256	8	16	1	≤ 0.06	128	0.125	0.25				
E12	16	8	4	>256	>256	>256	256	2	2	128	>256	0.5	0.25	A	NDM-5	ST410	UT/55
E12-J53	8	4	8	>256	>256	>256	32	2	0.5	≤ 0.06	256	0.5	0.25				
E22	>32	24	>32	>256	>256	>256	>256	4	2	64	>256	0.5	1	B	NDM-5	ST617	X3/55
E22-J53	8	2	6	>256	>256	>256	32	1	1	≤ 0.06	>256	0.25	0.5				
E21	>32	12	>32	>256	>256	>256	128	>256	4	1	>256	0.5	0.5	B	NDM-5	ST155	X3/55
E21-J53	16	6	8	>256	>256	>256	16	32	2	≤ 0.06	256	0.5	0.25				
E28	>32	>32	>32	>256	>256	>256	>256	>256	128	64	256	0.5	0.5	B	NDM-5	ST167	X3/55
E28-J53	16	4	8	>256	>256	>256	32	16	0.5	≤ 0.06	256	0.125	0.5				
E36	>32	>32	>32	>256	>256	>256	256	1	4	64	>256	0.25	0.25	C	NDM-5	ST2659	FI/55
E36-J53	8	2	4	>256	>256	>256	64	2	1	≤ 0.06	>256	0.25	< 0.125				
E37	>32	>32	>32	>256	>256	>256	256	1	2	128	>256	0.5	1	C	NDM-5	ST156	X3/55
E37-J53	8	2	4	>256	>256	>256	32	2	1	≤ 0.06	256	0.25	0.25				
E49	>32	>32	>32	>256	>256	>256	>256	>256	2	256	>256	0.125	0.5	D	NDM-5	ST167	X3/55
E49-J53	16	6	8	>256	>256	>256	32	128	0.5	≤ 0.06	>256	0.125	0.5				
E33	>32	>32	>32	>256	>256	>256	256	>256	>256	128	128	0.5	0.5	D	NDM-5	ST405	FI/55
E33-J53	4	2	2	>256	>256	>256	16	1	32	≤ 0.06	>256	0.25	0.125				
E47	>32	>32	>32	>256	>256	>256	256	4	8	8	>256	0.25	0.5	E	NDM-5	ST410	UT/55
E47-J53	8	4	6	>256	>256	>256	16	2	0.5	≤ 0.06	>256	0.25	0.5				
E48	>32	>32	>32	>256	>256	>256	256	4	4	128	>256	0.5	0.5	E	NDM-5	ST2083	FI/55
E48-J53	4	2	3	>256	>256	>256	16	1	0.5	≤ 0.06	>256	0.125	0.5				
E15	>32	8	8	>256	>256	>256	>256	>256	2	64	>256	0.25	0.25	A	NDM-1	ST167	FII/210
E15-J53	8	4	4	>256	>256	>256	32	2	0.25	≤ 0.06	>256	0.25	< 0.125				
E3	32	4	8	>256	>256	>256	128	256	4	64	>256	0.25	0.125	A	NDM-1	ST405	X3/55
E3-J53	12	4	4	>256	>256	>256	16	>256	2	≤ 0.06	>256	0.25	< 0.125				
E20	>32	>32	>32	>256	>256	>256	128	256	2	256	>256	0.25	0.5	B	NDM-1	ST410	X3/55
E20-J53	8	4	4	>256	>256	>256	128	256	0.25	≤ 0.06	>256	0.25	0.125				
E8	>32	8	8	>256	>256	>256	>256	256	2	128	>256	0.5	0.5	B	NDM-1	ST167	X3/210
E8-J53	16	4	8	>256	>256	>256	16	256	1	≤ 0.06	>256	0.5	0.25				
E44	>32	12	12	>256	>256	>256	64	1	2	256	128	0.125	0.25	C	NDM-1	ST167	X3/170
E44-J53	16	2	4	>256	>256	>256	32	>256	0.5	≤ 0.06	128	0.125	0.25				
E32	>32	>32	>32	>256	>256	>256	256	256	4	256	>256	0.5	1	D	NDM-1	ST167	FI/55
E32-J53	8	2	4	>256	>256	>256	16	2	0.5	≤ 0.06	256	0.125	0.125				
E53	16	8	6	>256	>256	>256	64	256	2	1	128	0.5	0.5	D	NDM-1	ST2376	X3/55
E53-J53	8	4	6	>256	>256	>256	16	1	0.25	≤ 0.06	128	0.5	0.25				
E6	16	8	8	>256	>256	>256	>256	>256	>256	64	>256	0.5	1	A	NDM-9	ST156	I1/105
E6-J53	6	2	2	>256	>256	>256	32	64	2	≤ 0.06	256	0.125	0.25				
E16	16	8	8	>256	>256	>256	128	>256	1	32	>256	0.25	0.25	A	NDM-4	ST410	X3/55
E16-J53	4	2	2	>256	>256	>256	16	1	0.5	≤ 0.06	>256	0.25	0.25				
E38	>32	>32	>32	>256	>256	>256	>256	>256	4	256	>256	0.125	0.5	C	NDM-7	ST410	FI/110
E38-J53	8	2	4	>256	>256	>256	16	4	2	≤ 0.06	256	0.125	0.125				
E39	>32	>32	>32	>256	>256	>256	256	>256	2	1	>256	0.5	0.5	C	NDM-7	ST167	X3/55
E39-J53	16	6	8	>256	>256	>256	32	128	1	≤ 0.06	256	0.25	0.25				
E41	>32	>32	>32	>256	>256	>256	256	>256	2	256	>256	0.25	1	C	NDM-7	ST2659	X3/55
E41-J53	8	4	6	>256	>256	>256	16	2	1	≤ 0.06	>256	0.25	0.25				
E45	>32	24	>32	>256	>256	>256	256	>256	>256	64	>256	0.5	0.5	E	NDM-7	ST617	X3/55
E45-J53	16	4	8	>256	>256	>256	16	256	2	≤ 0.06	>256	0.125	< 0.125				
E46	>32	12	>32	>256	>256	>256	>256	>256	>256	128	>256	0.5	0.25	E	NDM-7	ST617	X3/55
E46-J53	8	4	6	>256	>256	>256	16	64	0.5	≤ 0.06	>256	0.5	0.125				
E.coli J53	≤ 0.125	0.25	≤ 0.125	4	≤ 0.125	≤ 0.125	≤ 0.125	≤ 0.125	≤ 0.125	≤ 0.125	2	0.125	< 0.125				

IMP, imipenem; ETP, ertapenem; MEP, meropenem; PB, colistin; TGC, tigecycline; ATM, aztreonam; FOX, cefoxitin; FEP, cefepime; CAZ, ceftazidim; CRO, cefatriaxone; YZP, piperacillin/tazobactam; AMK, amikacin; CIP, ciprofloxacina: a

a *GenBank accession no. NC_022740.1*;

b *GenBank accession no. AP018144.1*.

**Figure 4:** Isolation and determination of plasmids harboring the *bla*_NDM_ gene in 26 clinical and transconjugants (**Top**: S1-nuclease PFGE patterns; **Bottom**: Southern blotting with a *bla*_NDM_ specific probe). The arrows represent thelocation of linear plasmid DNA hybridized with the *bla*_NDM_ specific probe. M: Braenderup H9812 Marker; lane 1: E5; lane 2: E7; lane 3: E12; lane4: E22; lane 5: E21; lane 6: E28; lane 7: E36; lane 8: E37; lane 9: E49; lane 10: E33; lane 11: E47; lane 12: E48; lane 13: E15; lane 14: E3; lane 15: E20; lane 16: E8; lane 17: E44; lane18: E32; lane 19: E53; lane 20: E6; lane 21: E16; lane 22: E38; lane 23: E39; lane 24: E41; lane 25: E45; lane 26: E46.

## Discussion

Metallo-lactamase, NDM, is an emerging carbapenem-resistant β-lactamase that is of major public concern due to its high medical and economic burden (Otter et al., 2017), especially for developing countries such as India, Pakistan, and the Balkan countries. As the most populous country in the world, there are major difficulties in preventing the dissemination of multidrug resistant genes in China. Therefore, comprehensive, extensive studies on diverse *bla*_NDM_ variant-positive *E. coli* are needed to provide clear information to optimize antibiotic policy in endemic areas.

Generally, the prevalence of the *bla*_NDM_ gene has continuously increased worldwide. As of now, the NDM enzyme has been identified in almost all of the world, including many countries in Asia, Africa, Europe, the Americas, and Australia (Berrazeg et al., 2014). A study from India also analyzed the occurrence of the *bla*_NDM_ gene among carbapenem resistant isolates, and it accounted for 45.4% of them (Rahman et al., 2018). Recently, a survey from the French National Reference Center revealed that among 140 carbapenem-resistant isolates 21% were NDM producer (Gauthier et al., 2018). In 2017, a nationwide study of clinical CRE strains in China demonstrated that 49% were NDM producer among carbapenem-resistant *E. coli* (Zhang et al., 2017). Furthermore, a multicenter study of the China CRE network revealed that among 39 carbapenem-resistant *E. coli* isolates, 74.4% were NDM producer, suggesting that there is a serious challenge in combating infections caused by this “superbug” in China (Zhang et al., 2018). In the present study, we identified 53 *bla*_NDM_-carrying isolates among 54 CRECO, which is much higher than in any other region of China (Wang S. et al., 2016; Hu et al., 2017; Liang et al., 2017). To the best of our knowledge, this is also the first report on the *bla*_NDM_ gene in Northern Jiangsu Province. Moreover, the emergence of such a high prevalence of *bla*_NDM_ variants indicates that the *bla*_NDM_ gene is increasing in this area.

Since its first identification in 2009, the *bl*a_NDM_ gene has evolved at a fast pace during the past 10 years. Twenty-one *bla*_NDM_ variants have been identified in different countries, all of which are archived at http://www.lahey.org/Studies/other.asp. Khan et al. (2017) reported that the Asian continent, especially China and India, was a reservoir of NDM producers, in which about a 58.2% abundance of the *bla*_NDM−1_ variants was found. Among these *bla*_NDM_ variants, the *bla*_NDM−1_ gene has been reported as the most prevalent type worldwide (Nordmann and Poirel, 2014). In our study, five *bla*_NDM_ variants were identified as responsible for MBL production, with the *bla*_NDM−5_ gene being the most prevalent. Compared with NDM-1, NDM-5 producers exhibited higher hydrolytic activity and toxicity toward carbapenem and cephalosporin (Mei et al., 2017). The *bla*_NDM−5_ gene is an emerging *bla*_NDM_ variants and has tended to surpass *bla*_NDM−1_ recently, and it differs from the NDM-1 enzyme at two amino acid substitutions, exhibited increased carbapenem resistance (Zhang et al., 2016). The *bla*_NDM−4_ and *bla*_NDM−7_ genes have been discovered among *E. coli* in China with relatively low prevalence, involving in 4 and 6 patients, respectively. Moreover, clinical *bla*_NDM−9_-positive *E. coli* has only been found in Taiwan (Lai et al., 2017), with this being the first report on the mainland China. Moreover, not merely NDM-5, amino acid substitutions in NDM-4 (M154L), NDM-7 (D130A), and NDM-9 (E152A) could also result in high levels of carbapenem resistance (Düzgün, 2018). Stewart et al. (2017) reported that the substitution in M154L, which is found in most *bla*_NDM_ variants, could enhance resistance to ampicillin at low zinc(II) concentrations relevant to infection sites.

*bla*_NDM_ variant-positive isolates exhibited multi-drug resistance. Variable resistances to aztreonam, amikacin, and ciprofloxacin were identified in NDM-1 and NDM-5-producing *E. coli*. The NDM-7, NDM-4, and NDM-9-producing isolates exhibited pan-resistant phenotypes, showing resistance to almost all commonly used clinical antibiotics except for colistin and tigecycline. In view of this, the expert recommended polymyxins was regarded as the last resort for NDM-producing isolates (Yamamoto and Pop-Vicas, 2014).

ST167 was confirmed as significant carrier in the present study, and is reported to be associated with the production of the NDM enzyme, especially NDM-5 (Chen et al., 2016). Notably, four *bla*_NDM_-positive ST617 strains were identified in the world, but we identified 6 isolates in the present study. Moreover, a novel new variant of *bla*_NDM_, *bla*_NDM−21_, belonged to ST617, which should deserve more attention (Liu et al., 2018). Furthermore, four new STs ST361, ST46, ST2376, and ST2083 were firstly reported to be linked with NDM-producing isolates.

The high efficiency of transfer renders the NDM producer ubiquitous throughout the world. Torres-González et al. (2015) reported an outbreak caused by *bla*_NDM−1_-carrying plasmid, which is easily transferred between *E. coli* and *Klebsiella pneumoniae*. Similarly, in the present study, the plasmids of 26 selected CRECO isolates were also tested for transfer. All selected *bla*_NDM−5_ genes were identified to be located on 55 kb plasmid, among which IncX3 was the most common replicon type. Notably, *bla*_NDM−5_ gene was frequently reported to be carried by the IncX3 plasmid of 55 kb in size, which was widely reported in China (Yang et al., 2014), Inidia (Krishnaraju et al., 2015), Australia (Wailan et al., 2015), and Damark (Hammerum et al., 2015). Moreover, Li et al. (2018) reported that IncX3 type plasmids play an important role in the transmission of the *bla*_NDM−5_ gene in *Enterobacteriaceae* and this kind of plasmid occurred in different species. Further illustrated the challenge of preventing the dissemination of the *bla*_NDM−5_ gene. The widespread *bla*_NDM−1_-carrying plasmid has been found to be associated with multiple replicon types, including IncX3, IncF, and IncA/C etc. In agreement with previous studies (Göttig et al., 2013; Wang L. H. et al., 2016), four *bla*_NDM−7_-positive plasmids were identified as ~55 kb IncX3 type, while the *bla*_NDM−7_ gene was also detected in the IncFI plasmid, which have been identified in India (Rahman et al., 2014). As for *bla*_NDM−9_, to the best of our knowledge, this is the first report on ~105 kb IncI1 type plasmid harboring *bla*_NDM−9_ gene. Overall, most plasmids harboring *bla*_NDM_ variants were identified as 55 kb IncX3 types, hinting that amino acid mutations might occur in the process of plasmid transfer, resulting in the emergence of *bla*_NDM_ variants. The high prevalence of the *bla*_NDM_ genes due in part to plasmid transfer, meanwhile, the fast evolution of this multidrug resistance gene also favors the persistence of such bacteria harboring it.

In summary, the present study reported high prevalence of *bla*_NDM_ variants, especially *bla*_NDM−5_, among carbapenem-resistant *E. coli* in Northern Jiangsu Province. The presence of five different variants further increases the threat to public health because of the limited treatment options. Notably, diverse *bla*_NDM_ variants were mainly located on ~55 kb IncX3 plasmids, indicating that the fast evolution and high transferability of this kind of plasmid has led to the high prevalence of *bla*_NDM_ variants. Timely detection of NDM enzyme and antimicrobial susceptibility testing are necessary so that infections caused by NDM producers receive appropriate and effective therapy. Similarly, large-scale surveillance and effective infection control measures are also urgently needed to prevent diverse *bla*_NDM_ variants from becoming epidemics in the future.

## Author contributions

The laboratory measurements were performed by RB, ZK, and HQ. BG and PM participated in experimental design and manuscript revision. Data analysis were implemented by RB, ZK, HQ, FJ, and HK.

### Conflict of interest statement

The authors declare that the research was conducted in the absence of any commercial or financial relationships that could be construed as a potential conflict of interest.

## References

[B1] Al-AgamyM. H.JeannotK.El-MahdyT. S.ShiblA. M.KattanW.PlésiatP.. (2017). First detection of GES-5 carbapenemase-producing *Acinetobacter baumannii* isolate. Microb. Drug Resist. 23, 556–562. 10.1089/mdr.2016.015227854148

[B2] AlbigerB.GlasnerC.StruelensM. J.GrundmannH.MonnetD. L. (2015). Carbapenemase-producing Enterobacteriaceae in Europe: assessment by national experts from 38 countries, May 2015. Euro. Surveill. 20:30062. 10.2807/1560-7917.ES.2015.20.45.3006226675038

[B3] BerrazegM.DieneS.MedjahedL.ParolaP.DrissiM.RaoultD. (2014). New Delhi Metallo-beta-lactamase around the world: an eReview using Google Maps. Euro. Surveill. 19:20809.2487175610.2807/1560-7917.es2014.19.20.20809

[B4] CarattoliA.BertiniA.VillaL.FalboV.HopkinsK. L.ThrelfallE. J. (2005). Identification of plasmids by PCR-based replicon typing. J. Microbiol. Methods 63, 219–228. 10.1016/j.mimet.2005.03.01815935499

[B5] ChenD.GongL.WalshT. R.LanR.WangT.ZhangJ.. (2016). Infection by and dissemination of NDM-5-producing *Escherichia coli* in China. J. Antimicrob. Chemother. 71, 563–565. 10.1093/jac/dkv35226542305

[B6] ChenY.ZhouZ.JiangY.YuY. (2011). Emergence of NDM-1-producing *Acinetobacter baumannii* in China. J. Antimicrob. Chemother. 66, 1255–1259. 10.1093/jac/dkr08221398294

[B7] Clinical and Laboratory Standards Institute [CLSI] (2017). Performance Standards for antimicrobial Susceptibility Testing, 27th Informational Supplement. Wayne, PA: Clinical and Laboratory Standards Institute.

[B8] DüzgünA. Ö. (2018). Effect of amino acid substitution in New Delhi metallo-β-lactamase on carbapenem susceptibility. Acta Microbiol. Immunol. Hung. 13, 1–9. 10.1556/030.65.2018.02229651859

[B9] EndimianiA.CariasL. L.HujerA. M.BethelC. R.HujerK. M.PerezF.. (2008). Presence of plasmid-mediated quinolone resistance in *Klebsiella pneumoniae* isolates possessing blaKPC in the United States. Antimicrob. Agents Chemother. 52, 2680–2682. 10.1128/AAC.00158-0818426899PMC2443894

[B10] GauthierL.DortetL.CotellonG.CretonE.CuzonG.PontiesV.. (2018). Diversity of Carbapenemase-producing *Escherichia coli* isolates in France in 2012-2013. Antimicrob Agents Chemother. 62:e00266–18. 10.1128/AAC.00266-1829866863PMC6105832

[B11] GöttigS.HamprechtA. G.ChristS.KempfV. A.WichelhausT. A. (2013). Detection of NDM-7 in Germany, a new variant of the New Delhi metallo-β-lactamase with increased carbapenemase activity. J. Antimicrob. Chemother. 68, 1737–1740. 10.1093/jac/dkt08823557929

[B12] HammerumA. M.HansenF.OlesenB.StruveC.HolzknechtB. J.AndersenP. S.. (2015). Investigation of a possible outbreak of NDM-5-producing ST16 *Klebsiella pneumoniae* among patients in Denmark with no history of recent travel using whole-genome sequencing. J. Glob. Antimicrob. Resist. 3, 219–221. 10.1016/j.jgar.2015.05.00327873714

[B13] HuX.XuX.WangX.XueW.ZhouH.ZhangL.. (2017). Diversity of New Delhi metallo-beta-lactamase-producing bacteria in China. Int. J. Infect. Dis. 55, 92–95. 10.1016/j.ijid.2017.01.01128104504

[B14] JinY.ShaoC.LiJ.FanH.BaiY.WangY. (2015). Outbreak of multidrug resistant NDM-1-producing *Klebsiella pneumoniae* from a neonatal unit in Shandong Province, China. PLoS ONE 10:e0119571. 10.1371/journal.pone.011957125799421PMC4370709

[B15] JohnsonT. J.BielakE. M.FortiniD.HansenL. H.HasmanH.DebroyC.. (2012). Expansion of the IncX plasmid family for improved identification and typing of novel plasmids in drug-resistant Enterobacteriaceae. Plasmid 68, 43–50. 10.1016/j.plasmid.2012.03.00122470007

[B16] KaaseM.NordmannP.WichelhausT. A.GatermannS. G.BonninR. A.PoirelL. (2011). NDM-2 carbapenemase in *Acinetobacter baumannii* from Egypt. J. Antimicrob. Chemother. 66, 1260–1262. 10.1093/jac/dkr13521427107

[B17] KhanA. U.MaryamL.ZarrilliR. (2017). Structure, genetics and worldwide spread of New Delhi Metallo-β-lactamase (NDM): a threat to public health. BMC Microbiol. 17:101. 10.1186/s12866-017-1012-828449650PMC5408368

[B18] KrishnarajuM.KamatchiC.JhaA. K.DevasenaN.VennilaR.SumathiG.. (2015). Complete sequencing of an IncX3 plasmid carrying blaNDM-5 allele reveals an early stage in the dissemination of the blaNDM gene. Indian J. Med. Microbiol. 33, 30–38. 10.4103/0255-0857.14837325559999

[B19] LaiC. C.ChuangY. C.ChenC. C.TangH. J. (2017). Coexistence of MCR-1 and NDM-9 in a clinical carbapenem-resistant *Escherichia coli* isolate. Int. J. Antimicrob. Agents 49, 517–518. 10.1016/j.ijantimicag.2017.02.00128219753

[B20] Leverstein-VanH. M. A.StuartJ. C.VoetsG. M.VersteegD.TersmetteT.FluitA. C. (2010). Global spread of New Delhi metallo-β-lactamase 1. Lancet Infect. Dis. 10, 830–831. 10.1016/S1473-3099(10)70277-221109170

[B21] LiX.FuY.ShenM.HuangD.DuX.HuQ.. (2018). Dissemination of blaNDM-5 gene via an IncX3-type plasmid among non-clonal *Escherichia coli* in China. Antimicrob. Resist. Infect. Control 7:59. 10.1186/s13756-018-0349-629713466PMC5918551

[B22] LiangW. J.LiuH. Y.DuanG. C.ZhaoY. X.ChenS. Y.YangH. Y.. (2017). Emergence and mechanism of carbapenem-resistant *Escherichia coli* in Henan, China, 2014. J. Infect. Public Health 11, 347–351. 10.1016/j.jiph.2017.09.02029107607

[B23] LiuL.FengY.McNallyA.ZongZ. (2018). blaNDM-21, a new variant of blaNDM in an *Escherichia coli* clinical isolate carrying blaCTX-M-55 and rmtB. J. Antimicrob. Chemother. 73, 2336–2339. 10.1093/jac/dky22629912337

[B24] MeiY. F.LiuP. P.WanL. G.LiuY.WangL. H.WeiD. D.. (2017). Virulence and genomic feature of a virulent *Klebsiella pneumoniae* sequence type 14 strain of serotype K2 harboring blaNDM-5 in China. Front. Microbiol. 8:335. 10.3389/fmicb.2017.0033528386246PMC5362587

[B25] NordmannP.PoirelL. (2014). The difficult-to-control spread of carbapenemase producers among Enterobacteriaceae worldwide. Clin. Microbiol. Infect. 20, 821–830. 10.1111/1469-0691.1271924930781

[B26] OtterJ. A.BurgessP.DaviesF.MookerjeeS.SingletonJ.GilchristM.. (2017). Counting the cost of an outbreak of carbapenemase-producing Enterobacteriaceae: an economic evaluation from a hospital perspective. Clin. Microbiol. Infect. 23, 188–196. 10.1016/j.cmi.2016.10.00527746394

[B27] PereiraP. S.BorghiM.de AraújoC. F.AiresC. A.OliveiraJ. C.AsensiM. D.. (2015). Clonal Dissemination of OXA-370-producing *Klebsiella pneumoniae* in Rio de Janeiro, Brazil. Antimicrob. Agents Chemother. 59, 4453–4456. 10.1128/AAC.04243-1425987619PMC4505195

[B28] Pérez-PérezF. J.HansonN. D. (2002). Detection of plasmid-mediated AmpC beta-lactamase genes in clinical isolates by using multiplex PCR. J. Clin. Microbiol. 40, 2153–2162. 10.1128/JCM.40.6.2153-2162.200212037080PMC130804

[B29] PoirelL.HéritierC.TolünV.NordmannP. (2004). Emergence of oxacillinase-mediated resistance to imipenem in *Klebsiella pneumoniae*. Antimicrob. Agents Chemother. 48, 15–22. 10.1128/AAC.48.1.15-22.200414693513PMC310167

[B30] QueenanA. M.Torres-VieraC.GoldH. S.CarmeliY.EliopoulosG. M.MoelleringR. C.. (2000). SME-type carbapenem-hydrolyzing class A beta-lactamases from geographically diverse *Serratia marcescens* strains. Antimicrob. Agents Chemother. 44, 3035–3039. 10.1128/AAC.44.11.3035-3039.200011036019PMC101599

[B31] RahmanM.MukhopadhyayC.RaiR. P.SinghS.GuptaS.SinghA.. (2018). Novel variant NDM-11 and other NDM-1 variants in multidrug-resistant *Escherichia coli* from South India. J. Glob. Antimicrob. Resist. 14, 154–157. 10.1016/j.jgar.2018.04.00129656053

[B32] RahmanM.ShuklaS. K.PrasadK. N.OvejeroC. M.PatiB. K.TripathiA.. (2014). Prevalence and molecular characterisation of New Delhi metallo-β-lactamases NDM-1, NDM-5, NDM-6 and NDM-7 in multidrug-resistant Enterobacteriaceae from India. Int. J. Antimicrob. Agents 44, 30–37. 10.1016/j.ijantimicag.2014.03.00324831713

[B33] SchmittJ.JacobsE.SchmidtH. (2007). Molecular characterization of extended-spectrum beta-lactamases in Enterobacteriaceae from patients of two hospitals in Saxony, Germany. J. Med. Microbiol. 56(Pt 2), 241–249. 10.1099/jmm.0.46670-017244807

[B34] SendaK.ArakawaY.IchiyamaS.NakashimaK.ItoH.OhsukaS.. (1996). PCR detection of metallo-beta-lactamase gene (blaIMP) in gram-negative rods resistant to broad-spectrum beta-lactams. J. Clin. Microbiol. 34, 2909–2913. 894042110.1128/jcm.34.12.2909-2913.1996PMC229432

[B35] StewartA. C.BethelC. R.VanPeltJ.BergstromA.ChengZ.MillerC. G.. (2017). Clinical variants of New Delhi metallo-β-lactamase are evolving to overcome zinc scarcity. ACS Infect. Dis. 3, 927–940. 10.1021/acsinfecdis.7b0012828965402PMC5726261

[B36] Torres-GonzálezP.Bobadilla-Del ValleM.Tovar-CalderónE.Leal-VegaF.Hernández-CruzA.Martínez-GamboaA.. (2015). Outbreak caused by Enterobacteriaceae harboring NDM-1 metallo-β-lactamase carried in an IncFII plasmid in a tertiary care hospital in Mexico City. Antimicrob. Agents Chemother. 59, 7080–7083. 10.1128/AAC.00055-15.26282410PMC4604355

[B37] WailanA. M.PatersonD. L.CafferyM.SowdenD.SidjabatH. E. (2015). Draft genome sequence of NDM-5-producing *Escherichia coli* sequence Type 648 and genetic context of blaNDM-5 in Australia. Genome. Announc. 3:e00194–15. 10.1128/genomeA.00194-1525858833PMC4392145

[B38] WalshT. R. (2010). Emerging carbapenemases: a global perspective. Int. J. Antimicrob. Agents 36(Suppl. 3), S8–S14. 10.1016/S0924-8579(10)70004-221129630

[B39] WangL. H.LiuP. P.WeiD. D.LiuY.WanL. G.XiangT. X.. (2016). Clinical isolates of uropathogenic *Escherichia coli* ST131 producing NDM-7 metallo-β-lactamase in China. Int. J. Antimicrob. Agents 48, 41–45. 10.1016/j.ijantimicag.2016.03.00927216384

[B40] WangS.ZhaoS. Y.XiaoS. Z.GuF. F.LiuQ. Z.TangJ.. (2016). Antimicrobial resistance and molecular epidemiology of *Escherichia coli* causing bloodstream infections in three hospitals in Shanghai, China. PLoS ONE 11:e0147740. 10.1371/journal.pone.014774026824702PMC4733056

[B41] WangX.XuX.LiZ.ChenH.WangQ.YangP.. (2014). An outbreak of a nosocomial NDM-1-producing *Klebsiella pneumoniae* ST147 at a teaching hospital in mainland China. Microb. Drug Resist. 20, 144–149. 10.1089/mdr.2013.010024199986

[B42] WirthT.FalushD.LanR.CollesF.MensaP.WielerL. H.. (2006). Sex and virulence in *Escherichia coli*: an evolutionary perspective. Mol. Microbiol. 60, 1136–1151. 10.1111/j.1365-2958.2006.05172.x16689791PMC1557465

[B43] YamamotoM.Pop-VicasA. E. (2014). Treatment for infections with carbapenem-resistant Enterobacteriaceae: what options do we still have? Crit. Care 18:229. 10.1186/cc1394925041592PMC4075344

[B44] YangJ.ChenY.JiaX.LuoY.SongQ.ZhaoW.. (2012). Dissemination and characterization of NDM-1-producing *Acinetobacter pittii* in an intensive care unit in China. Clin. Microbiol. Infect. 18, E506–E513. 10.1111/1469-0691.1203523036089

[B45] YangP.XieY.FengP.ZongZ. (2014). blaNDM-5 carried by an IncX3 plasmid in *Escherichia coli* sequence type 167. Antimicrob. Agents Chemother. 58, 7548–7552. 10.1128/AAC.03911-1425246393PMC4249565

[B46] YongD.TolemanM. A.GiskeC. G.ChoH. S.SundmanK.LeeK.. (2009). Characterization of a new metallo-beta-lactamase gene, bla(NDM-1), and a novel erythromycin esterase gene carried on a unique genetic structure in *Klebsiella pneumoniae* sequence type 14 from India. Antimicrob. Agents Chemother. 53, 5046–5054. 10.1128/AAC.00774-0919770275PMC2786356

[B47] YuJ.TanK.RongZ.WangY.ChenZ.ZhuX.. (2016). Nosocomial outbreak of KPC-2- and NDM-1-producing *Klebsiella pneumoniae* in a neonatal ward: a retrospective study. BMC Infect. Dis. 16:563. 10.1186/s12879-016-1870-y27733128PMC5062924

[B48] YuY.JiS.ChenY.ZhouW.WeiZ.LiL.. (2007). Resistance of strains producing extended-spectrum beta-lactamases and genotype distribution in China. J. Infect. 54, 53–57. 10.1016/j.jinf.2006.01.01416533535

[B49] ZhangF.XieL.WangX.HanL.GuoX.NiY. (2016). Further spread of blaNDM-5 in Enterobacteriaceae via IncX3 plasmids in Shanghai, China. Front. Microbiol. 7:424 10.3389/fmicb.2016.0042427065982PMC4811927

[B50] ZhangR.LiuL.ZhouH.ChanE. W.LiJ.FangY.. (2017). Nationwide surveillance of clinical Carbapenem-resistant Enterobacteriaceae (CRE) strains in China. EBioMedicine 19, 98–106. 10.1016/j.ebiom.2017.04.03228479289PMC5440625

[B51] ZhangY.WangQ.YinY.ChenH.JinL.GuB.. (2018). Epidemiology of carbapenem-resistant Enterobacteriaceae infections: report from the China CRE network. Antimicrob. Agents Chemother. 62. 10.1128/AAC.01882-1729203488PMC5786810

[B52] ZilberbergM. D.ShorrA. F. (2013). Secular trends in gram-negative resistance among urinary tract infection hospitalizations in the United States, 2000-2009. Infect. Control Hosp. Epidemiol. 34, 940–946. 10.1086/67174023917908

